The article "Association between the Length of Hospital Stay and 30-Day Outcomes in Patients Admitted with Acute Decompensated Heart Failure" was published in 2023. Journal: Emerg Med Int.

# Association between the Length of Hospital Stay and 30-Day Outcomes in Patients Admitted with Acute Decompensated Heart Failure

**DOI:** 10.1155/2023/6338597

**Published:** 2023-03-06

**Authors:** Melika Namvar, Mohammad Fakhrolmobasheri, Sadegh Mazaheri-Tehrani, Maryam Heidarpour, Maryam Emamimeybodi, Davood Shafie

**Affiliations:** ^1^Heart Failure Research Center, Isfahan Cardiovascular Research Institute, Isfahan University of Medical Sciences, Isfahan, Iran; ^2^Student Research Committee, School of Medicine, Isfahan University of Medical Sciences, Isfahan, Iran; ^3^Isfahan Endocrine and Metabolism Research Center, Isfahan University of Medical Sciences, Isfahan, Iran; ^4^UCLA Cardiac Arrhythmia Center, University of California, Los Angeles, California, USA; ^5^UCLA Neurocardiology Program of Excellence, University of California, Los Angeles, California, USA

## Abstract

**Method:**

This study is performed in the context of the Persian Registry of Cardiovascular Disease/Heart Failure (PROVE/HF). We included all patients admitted with ADHF regardless of the etiology of heart failure (HF). LOS was classified in tertiles (<4 days, >4 and <6 days, and >6 days). Our outcomes were 30-day all-cause mortality and rehospitalization. Baseline characteristics and outcomes are reported according to the tertiles of LOS. A binary logistic regression and cox regression analysis were performed to evaluate the association between LOS and rehospitalization and death, respectively.

**Results:**

Between April 2019 and March 2020, 385 patients with ADHF were registered in our study. The mean length of hospitalization was 6.35 ± 5.46 days, varying from a minimum of 0 days to a maximum of 47 days. One hundred patients had a hospital stay lower than 4 days; 151 individuals had an intermediate LOS (4–6 days); and 134 were hospitalized for more than 6 days. Our analysis indicated no association between LOS and 30-day rehospitalization and death in multivariable or univariable models.

**Conclusion:**

This study found no association between LOS and rehospitalization or death in patients admitted with ADHF; however, further investigations are warranted.

## 1. Introduction

Heart failure (HF) is a global health concern with an increasing number of individuals older than 50 years. The global prevalence of HF is reported to be 64.34 million cases [1], and it is one of the major causes of hospitalization (over 1 million patients annually) in the USA [2]. The total medical costs for HF patients are expected to reach US$53.1 billion by 2030 [3]. Acute decompensated heart failure (ADHF) is a condition in which patients suffer from a rapid worsening of HF signs and symptoms [4]. Most patients (80%) hospitalized due to HF present as ADHF [5, 6].

Investigations suggest that hospital length of stay (LOS) may be a valuable predictor of outcomes for patients hospitalized for ADHF, including rates of early readmission and mortality. On the other hand, other factors, including peripheral edema, chest pain, elevated jugular venous pressure, increased weight during hospitalization, anemia, renal insufficiency, and diuretic dose at admission, as well as some laboratory parameters such as serum albumin, sodium, creatinine, and cardiac troponin level are reported to be associated with longer LOS in patients with ADHF [7–10]. Accordingly, the inflammatory status and severity of congestion at admission have been reported to be key factors in predicting the LOS in ADHF [11]. Recent studies indicated conflicting results regarding the LOS of HF patients and the rate of readmission or mortality [12–15]. It is notable that patients who survive an ADHF event are at a considerably higher risk for the incidence of cardiovascular events during the first month postdischarge [16]. Studies suggested that countries with longer LOS for HF hospitalization had significantly lower rates of 30-day readmission [17], along with the results of a multinational cohort study [18]. In contrast, other studies found that short and long LOS were associated with a higher risk of readmission and even greater overall costs among HF patients [15, 17, 19].

Regarding the controversial reports surrounding the association of LOS with the outcomes of patients with ADHF and the heterogeneity among the healthcare policies in different regions [20], we conducted a retrospective study on the patient from the Persian Registry of Cardiovascular Disease–Heart Failure (PROVE/HF) to better indicate the association of LOS with the outcomes of patients, particularly in the setting of our regional healthcare policies. Furthermore, we attempted to evaluate the factors that might affect the length LOS including the medications administered during hospitalization and the patients' inflammatory and hemodynamic status at admission. Regarding inflammatory status, we used the neutrophil to lymphocyte ratio (NLR), platelets to lymphocyte ratio (PLR), and red cell distribution width (RDW) as markers of systemic inflammation and modified shock index (MSI) as a marker of hemodynamic instability [21–24].

## 2. Method

### 2.1. Study Design and Participants

This retrospective cohort study was conducted in the context of the Persian Registry of Cardiovascular Disease/Heart Failure (PROVE/HF) database, launched in March 2015, and continuously gathering data on HF patients admitted to Chamran Cardiology Hospital, Isfahan, Iran, with the primary diagnosis of ADHF. Detailed information regarding the methodology of the PROVE/HF study is reported separately [25]. From April 2019 to March 2020, any individual aged at least 18 years suffering from ADHF admitted to the tertiary governmental heart center (Charman hospital, Isfahan, Iran) was eligible for inclusion in our study. We included those patients admitted to the emergency department. All patients with previously proven HF who were referred with signs and symptoms of decompensation had an equal chance to be included. Patients with untreated chronic complications, including severe liver diseases, malignancy, severe infection, current usage of chemotherapeutic drugs, unwillingness to participate in the study, or incompleteness of their medical profiles, were excluded. We further excluded admitted HF individuals with stable conditions including patients admitted to the echocardiography ward, patients referred for electrophysiological study and device implantation, and patients admitted for elective coronary evaluation or valvular interventions. Each participant was fully informed of the aims of the study. This study was approved by the ethics committee of the Isfahan University of Medical Sciences.

### 2.2. Study Outcomes

The primary outcomes of the PROVE/HF were rehospitalization and death due to acute decompensated heart failure. Secondary outcomes included all-cause death and rehospitalization.

### 2.3. Data Collection

Using a predefined questionnaire all demographic characteristics and past medical history of participants, including age, gender (male/female), body mass index (BMI), smoking status (%), blood pressure (BP) indices including systolic BP (SBP) and diastolic BP (DBP), LOS (day), heart rate, ischemic heart disease (%), diabetes mellitus (%), hypertension (%), kidney diseases (%), and thyroid disorders (%). Laboratory parameters, including hemoglobin (g/dL), sodium (mEq/L), potassium (mEq/L), blood urea nitrogen (mg/dL), and creatinine (mg/dL), were measured at admission time through blood samples. Moreover, all participants were asked for the consumption of different drugs, including beta blockers, angiotensin-converting enzyme inhibitors (ACEIs), angiotensin receptor blockers (ARBs), mineralocorticoid receptor antagonists (MRA), and diuretics. Left ventricular ejection fraction (LVEF) was also recorded from the echocardiography report in the current hospitalization.

### 2.4. Follow-Up Surveys

All of the surviving participants were followed up at 1^st^, 6^th^, and 12^th^ month after discharge through telephone call interviews. The telephone follow-ups were performed by trained staff using a predefined questionnaire. In any case of uncertainty or failure to obtain proper information through a telephone interview, the patients or the patients' relatives were appointed for a face-to-face interview with a cardiologist. Regarding outcome adjudication, proper documentation was requested from patients/first-degree relatives in terms of death or rehospitalization, and if the documentations were of any uncertainty, an outcome adjudication panel reviewed all the available documents associated with the outcomes of interest.

### 2.5. Factors Associated with LOS

A modified shock index was calculated by dividing heart rate over mean arterial pressure (MAP). PLR was calculated as platelet counts divided by the absolute lymphocyte count. NLR was calculated as absolute neutrophil count divided by the lymphocyte count. RDW-CV (RDW- coefficient of variation) was calculated as RDW-CV = (standard deviation of MCV ÷ MCV) × 100.

### 2.6. Statistical Analysis

Continuous variables are reported as the mean ± standard deviation. Categorical variables are presented as number and frequency. Between-group differences were assessed by ANOVA and chi-square tests for continuous and categorical variables, respectively. Odds ratios were obtained by binary logistic regression analysis. Hazard ratios were obtained using cox regression analysis. Multivariable regression analysis was performed using confounding variables with statistically significant association with the outcomes identified by stepwise backward regression analysis.

## 3. Result

Between April 2019 and March 2020, 385 patients with ADHF were registered in our study. The mean age of participants was 66.13 ± 13.2 years, and 66.5% of patients were men. The mean length of hospitalization was 6.35 ± 5.46 days, varying from a minimum of 0 days to a maximum of 47 days. The LOS of participants was divided into three groups: 100 patients had a hospital stay lower than 4 days, 151 individuals had an intermediate LOS (4–6 days), and 134 patients were hospitalized for more than 6 days.  Table 1 categorized participants' baseline characteristics and drug history according to LOS. There are significant differences in serum creatinine and hemoglobin levels within LOS tertiles.

The distribution of 30-day readmission and mortality among different tertiles of LOS is shown in Table 2. According to follow-up documents, rehospitalization and mortality rates among participants were 26% and 13%, respectively. Rehospitalization and death among the study population did not show significant differences within different groups of hospitalized patients. Due to binary logistic regression, there is no significant association between rehospitalization rate and duration of hospital stay. Results remain insignificant even after adjustment for baseline characteristics (Table 3). The hazard ratio of death according to LOS is shown in Table 4. There is a significant association between longer LOS and mortality rate in the crude model, but after adjustment with baseline characteristics, the results became insignificant.

### 3.1. Length of Hospital Stay among Subtypes of HF

As demonstrated in Table 1 there is no significant difference among the number of patients with different types of HF in the tertiles of LOS; however, the mean ± SD of LOS was significantly higher in patients with HFmrEF but in line with findings in Table 1, there was no difference in LOS between HFrEF and HFpEF patients (Table 5).

### 3.2. Factors Associated with LOS

Table 5 demonstrate the mean ± SD of NLR, PLR, MSI, and RDW-CV divided by the subtypes of HF. We did not observe any difference in the abovementioned markers among the HF subgroup. On the other hand, when comparing the mean of inflammatory markers among the tertiles of LOS, we observed that the NLR was significantly higher in participants with higher LOS (Table 6). Furthermore, in Tables 7 and 8 we compared the mean ± SD of inflammatory markers and MSI among tertiles of LOS divided the subgroups of HF (HFrEF vs. HFpEF and HFmrEF). Interestingly, we observed that in HFpEF and HFmrEF patients, NLR was significantly higher in patients with higher LOS but in patients with HFrEF none of the inflammatory markers or MSI were significantly different among the tertiles of LOS. Regarding the treatments during the hospitalization, as summarized in Table 9, only administration of inotrope drugs was prognostic for higher LOS.

## 4. Discussion

In this retrospective cohort study of 385 participants with ADHF, 100 patients were readmitted to the hospital within 30 days, and 50 died during follow-up after discharge. The mean length of hospitalization was 6.35 ± 5.46 days. According to recent studies, the LOS of HF patients varies in different regions. The median LOS in the US and Europe was 6 and 9 days, respectively [26, 27]. While in Japan, the ATTEND and JCARE-CARD registries reported the median LOS of HF patients 21 and 15 days, respectively [28, 29]. Differences among local medical practices and healthcare systems might be the reason for this variation [15]. In this regard, the LOS of HF patients was categorized differently in studies. We classify the LOS of our patients into three groups: less than 4 days (short LOS), 4–6 days (intermediate LOS), and more than 6 days (prolonged LOS).

There is no significant association between LOS and the 30-day readmission rate, even after adjustment with baseline features. Recently, 30-day readmission was demonstrated to be a good indicator of hospital performance [30]. Up to now, studies have also indicated various results. Khan et al. [18] showed that longer LOS was associated with a lower risk of readmissions due to HF, while Sud et al. [31] revealed that longer LOS for HF was associated with a higher risk of HF readmissions. They also showed that short LOS was associated with an increased risk of HF readmissions, the same as the results of another cohort study in Japan [15]. However, Reynolds et al. [12] did not find a significant association between short LOS and readmission within 30 days. A retrospective observational study by Kociol et al. [30] reported the same results as ours. The authors had postulated that the LOS would not be associated with the 30-day readmission rate. Moreover, they reported the mean days of hospital stay as 4.9 (4.2–5.6). These results are consistent with our reported mean number of days for the hospital stay.

The hazard ratio of death among participants after discharge was significant only within the long LOS and short LOS groups before adjustment for baseline characteristics, showing that longer than 6-day hospitalization might cause a higher mortality rate after discharge, which might be related to the poor prognosis of ADHF patients [20]. Recent research has also demonstrated a higher mortality risk among patients with longer LOS [12, 13, 20, 31].

Anemia is a common complication among ADHF patients, and studies have demonstrated its association with longer LOS and an even higher rate of mortality and rehospitalization [9, 32–35]. In the current study, patients with longer LOS reported lower hemoglobin levels. However, a population-based study in Spain did not find significant differences between long and short LOS [36].

Higher baseline serum creatinine levels of ADHF patients are an indicator for the subgroup of patients with the possibility of a longer LOS [36]. Our results also demonstrated a higher baseline creatinine level in patients with longer LOS. Recent studies have indicated that systemic inflammation and the severity of congestion are strong predictors of LOS. Regarding congestion, several indicators have been proposed to be indicative of the severity of congestion including ultrasound-guided evaluation of lung congestion, renal venous flow, vena cava, and right heart function [37, 38]. Nevertheless, in this study, we were not able to assess the aforementioned indicators of congestion, thus, we tend to use MSI as an indicator of hemodynamic instability which could be indirectly associated with a severity of congestion; however, we failed to find any significant association between MSI and LOS [23]. In line with congestion, systemic inflammation is reported to be a predictor of LOS, particularly in patients with HFpEF [11]. As postulated by Pugliese et al., inflammatory factors such as Galectin-3, InterLeukin-1, and several other immunologic markers may be indicative for inflammation in ADHF but unfortunately, in this study, we were not able to measure the above mentioned markers; however, we use NLR, PLR, and RDW as indirect markers of inflammation in HF [21, 22, 24]. Accordingly, we have observed that NLR was significantly higher in HFpEF patients with higher LOS; however, in patients with HFrEF, it was not associated with higher LOS.

Our study has several limitations. First, patients are discharged due to the clinician's decision, so their condition at the time of discharge was not the same in different cases. Second, according to recent reports, several other factors might be associated with LOS, such as socioeconomic status, hospital environment, treatment staff, and self-care behavior [15]. Third, we calculate only the readmissions due to HF. Therefore, we cannot determine whether there is a relationship between LOS and readmissions for other reasons. We are the first group assessing the effect of LOS in ADHF patients with hospital readmission and mortality in Isfahan, so further studies in different regions (e.g., rural areas) and other treatment centers will be needed to confirm our results.

## 5. Conclusion

Our results indicated no association between length of hospital stay and 30-day mortality and rehospitalization in patients with ADHF; however, these findings need to be further investigated since multiple factors may impact the outcomes in this group of patients.

## Figures and Tables

**Table 1:** General and laboratory characteristics and drug history of the study population according to the length of hospital stay.

Variables	Total (*n* = 385)	Length of hospital stay			*P* ^*∗*^
		<4 days (*n* = 100)	4–6 days (*n* = 151)	>6 days (*n* = 134)	
Age (years)	66.13 ± 13.20	65.05 ± 12.56	66.83 ± 13.14	66.15 ± 13.77	0.581
Males (%)	252 (65.5)	69 (69)	101 (66.9)	82 (61.2)	0.413
BMI (kg/m^2^)	27.10 ± 6.64	26.29 ± 4.09	27.70 ± 8.70	26.97 ± 5.34	0.229
Tachycardia (%)	75 (19.5)	27 (27)	22 (14.6)	26 (19.4)	0.052
Ischemic heart disease (%)	342 (88.8)	88 (88)	132 (87.4)	122 (91)	0.596
Diabetes mellitus (%)	168 (43.6)	33 (33)	69 (45.7)	66 (49.3)^a^	0.037
Hypertension (%)	194 (50.4)	48 (48)	78 (51.7)	68 (50.7)	0.847
Kidney diseases (%)	173 (44.9)	39 (39)	68 (45)	66 (49.3)	0.296
Thyroid disorders (%)	51 (13.2)	13 (13)	20 (13.2)	18 (13.4)	0.995
Anemia (%)	47 (12.2)	15 (15)	11 (7.3)	21 (15.7)	0.060
Smoking status (%)	136 (35.3)	42 (42)	59 (39.1)	35 (26.1)^a^	0.020
Systolic blood pressure (mmHg)	123.02 ± 24.95	125.78 ± 24.37	122.11 ± 23.47	121.99 ± 26.95	0.438
Diastolic blood pressure (mmHg)	76.55 ± 15.65	79.41 ± 16.27	75.21 ± 15.69	75.93 ± 14.97	0.098
Hemoglobin (g/dl)	13.43 ± 2.22	14.01 ± 2.22	13.55 ± 2.07^b^	12.88 ± 2.29^a^	<0.001
Sodium (mEq/l)	136.14 ± 4.48	136.62 ± 4.49	136.04 ± 4.33	135.90 ± 4.64	0.445
Potassium (mEq/l)	4.29 ± 0.58	4.26 ± 0.51	4.29 ± 0.59	4.31 ± 0.61	0.845
Blood urea nitrogen (mg/dl)	48.38 ± 18.29	45.99 ± 17.23	48.54 ± 18.13	49.97 ± 19.15	0.256
Creatinine (mg/dl)	1.49 ± 0.86	1.29 ± 0.43	1.54 ± 0.94	1.59 ± 0.99^a^	0.022
HF type					
HFrEF	304 (77.4%)	77 (77.0%)	116 (76.8%)	105 (78.4%)	0.071
HFmrEF	49 (12.5%)	7 (7.0%)	24 (15.9%)	17 (12.7%)	
HFpEF	40 (10.2%)	16 (16.0%)	11 (7.3%)	12 (9.0%)	
Discharge drug					
Beta-blockers (%)	292 (75.8)	79 (79)	116 (76.8)	97 (72.4)	0.473
ACEIs/ARBs (%)	320 (83.1)	84 (84)	127 (84.1)	109 (81.3)	0.794
Mineralocorticoid receptor antagonists (%)	113 (29.4)	27 (27)	51 (33.8)	35 (26.1)	0.306
Diuretics (%)	329 (85.5)	86 (86)	130 (86.1)	113 (84.3)	0.900

BMI, body mass index; ACEIs, angiotensin-converting enzyme inhibitors; ARBs, angiotensin receptor blockers; HF, heart failure; HFrEF, HF with reduced ejection fraction; HFmrEF, HF with mildly reduced ejection fraction; HFpEF, HF with preserved ejection fraction. ^*∗*^Results from One-Way ANOVA and chi-square test, as appropriate. a: *P* values <0.05 resulted from a comparison of hospital stay of >6 days vs. hospital stay of <4 days. b: *P* values <0.05 resulted from a comparison of hospital stay of >6 days vs. hospital stay of 4–6 days.

**Table 2:** Distribution of rehospitalization and death among the study population according to the length of hospital stay.

Variables	Total	Length of hospital stay			*P* ^*∗*^
		<4 days (*n* = 100)	4–6 days (*n* = 151)	>6 days (*n* = 134)	
Rehospitalization	100 (26)	29 (29)	41 (41)	30 (30)	0.477
Death	50 (13)	8 (16)	18 (36)	24 (48)	0.073

^*∗*^: resulted from chi-square test.

**Table 3:** Crude and adjusted odds ratio of rehospitalization according to the length of hospital stay.

Variable	Models	Length of hospital stay			*Pƪ*	*P*¶
		<4 days (*n* = 100)	4–6 days (*n* = 151)	>6 days (*n* = 134)		
Rehospitalization	Crude	1.00	1.09 (0.63–1.92)	1.42 (0.78–2.56)	0.749	0.250
	Adjusted^*∗*^	1.00	1.04 (0.57–1.88)	1.55 (0.82–2.95)	0.911	0.178

Binary Logistic Regression. ^*∗*^Adjusted for age, sex, body mass index, tachycardia, ischemic heart disease, diabetes mellitus, hypertension, kidney diseases, thyroid disorders, anemia, smoking status, systolic blood pressure, diastolic blood pressure, hemoglobin, sodium, potassium, blood urea nitrogen, creatinine, and before drug consumption (beta-blockers, angiotensin-converting enzyme inhibitors, angiotensin receptor blockers, mineralocorticoid receptor antagonists, and diuretics). *Pƪ*: *P* value resulted from a comparison between hospital stay of <4 days vs. hospital stay of 4–6 days. *P*¶: *P* value resulted from a comparison between hospital stay of <4 days vs. hospital stay of >6 days.

**Table 4:** Crude and adjusted cox regression hazard ratio of death according to the length of hospital stay.

Variables	Models	Length of hospital stay			*Pƪ*	*P*¶
		<4 days (*n* = 100)	4–6 days (*n* = 151)	>6 days (*n* = 134)		
Death	Crude	1.00	1.56 (0.67–3.61)	2.39 (1.06–5.37)	0.299	0.035
	Adjusted^*∗*^	1.00	0.91 (0.36–2.29)	1.51 (0.61–3.75)	0.848	0.377

^*∗*^Adjusted for age, sex, body mass index, tachycardia, ischemic heart disease, diabetes mellitus, hypertension, kidney diseases, thyroid disorders, anemia, smoking status, systolic blood pressure, diastolic blood pressure, hemoglobin, sodium, potassium, blood urea nitrogen, creatinine, and before drug consumption (beta-blockers, angiotensin-converting enzyme inhibitors, angiotensin receptor blockers, mineralocorticoid receptor antagonists, and diuretics). *Pƪ*: *P* value resulted from a comparison between hospital stay of <4 days vs. hospital stay of 4–6 days. *P*¶: *P* value resulted from a comparison between hospital stay of <4 days vs. hospital stay of >6 days.

**Table 5:** Length of hospital stay, neutrophil to lymphocyte ratio (NLR), platelets to lymphocyte ratio (PLR), modified shock index (MSI), rehospitalization and death during 30-days follow-up divided by the EF groups. ^*∗*^significant between group difference.

	EF groups		
	HFrEF	HFmrEF	HFpEF
	Mean (Standard deviation)/Number (Percentage)		
Length of hospital stay^*∗*^	**6 (5)**	**8 (9)**	**6 (7)**
NLR	4.17 (3.32)	4.31 (3.11)	4.11 (2.61)
PLR	134.70 (95.70)	138.87 (64.70)	122.38 (70.60)
MSI	0.95 (0.25)	0.95 (0.28)	0.90 (0.17)
Rehospitalization	73 (24.0%)	15 (30.6%)	12 (30.0%)
F/U death	38 (12.5%)	7 (14.3%)	5 (12.5%)

Bold values indicate values with significant differences among HF sub-types.

**Table 6:** Mean ± SD of neutrophil to lymphocyte ratio (NLR), platelets to lymphocyte ratio (PLR), modified shock index (MSI), and red cell distribution width (RDW) among the tertiles of hospitalization time in total study population. ^*∗*^significant between group difference.

	Length of hospital stay		
	<4	4–6	>6
	Mean (standard deviation)/Number (percentage)		
MSI	0.97 ± 0.27	0.93 ± 0.24	0.95 ± 0.25
PLR	117.70 ± 61.10	144.16 ± 107.49	136.03 ± 86.71
NLR^*∗*^	**3.51** **±** **2.88**	**4.19** **±** **2.72**	**4.54** **±** **3.67**
RDW_CV	15.7 ± 1.9	15.9 ± 2.4	16.2 ± 2.6

**Table 7:** Mean ± SD of neutrophil to lymphocyte ratio (NLR), platelets to lymphocyte ratio (PLR), modified shock index (MSI), and red cell distribution width (RDW) among the tetile of hospitalization time in patients with HFrEF. ^*∗*^significant between group difference.

	Length of hospital stay		
	<4	4–6	>6
	Mean (standard deviation)/number (percentage)		
MSI	0.98 (0.27)	0.92 (0.24)	0.96 (0.26)
PLR	121.42 (64.15)	143.94 (114.45)	136.67 (93.45)
NLR	3.72 (3.17)	4.15 (2.85)	4.43 (3.66)
RDW_CV	15.7 (2.0)	15.8 (2.3)	16.1 (2.5)

**Table 8:** Mean ± SD of neutrophil to lymphocyte ratio (NLR), platelets to lymphocyte ratio (PLR), modified shock index (MSI), and red cell distribution width (RDW) among the tertile of hospitalization time in patients with HFpEF and HFmrEF. ^*∗*^significant between group difference.

	Length of hospital stay		
	<4	4–6	>6
	Mean (Standard deviation)/Number (Percentage)		
MSI	0.94 (0.31)	0.94 (0.23)	0.90 (0.20)
PLR	105.25 (48.72)	144.87 (81.67)	133.73 (57.14)
NLR^*∗*^	**2.81 (1.36)**	**4.34 (2.27)**	**4.96 (3.76)**
RDW_CV	15.5 (1.4)	16.1 (2.5)	16.5 (2.7)

Bold values indicate values with significant differences among tertiles of length of hospital stay.

**Table 9:** Drugs administered for patients during hospitalization divided by the tertiles of LOS. ^*∗*^significant between group difference.

	Length of hospital stay		
	<4	4–6	>6
	Number (Percentage)		
ACEIs	48 (24.4%)	77 (39.1%)	72 (36.5%)
ARBs	44 (26.7%)	70 (42.4%)	51 (30.9%)
Beta blockers	84 (27.3%)	119 (38.6%)	105 (34.1%)
Diuretics	93 (26.1%)	137 (38.5%)	126 (35.4%)
MRAs	38 (25.2%)	63 (41.7%)	50 (33.1%)
Statins	55 (24.6%)	93 (41.5%)	76 (33.9%)
Inotropes^*∗*^	**5 (11.1%)**	**16 (35.6%)**	**24 (53.3%)**
Nitrates	6 (22.2%)	9 (33.3%)	12 (44.4%)
Aspirin	58 (26.5%)	83 (37.9%)	78 (35.6%)
ADP inhibitors	17 (21.5%)	33 (41.8%)	29 (36.7%)
PPIs	51 (23.5%)	89 (41.0%)	77 (35.5%)

ACEIs, angiotensin converting enzyme inhibitors; ARBs, angiotensin receptor blockers; MRAs, mineralocorticoid receptor antagonists; ADP inhibitors, adenosine diphosphate (ADP) receptor inhibitors; PPI, proton pump inhibitors. Bold values indicate values with significant differences among tertiles of length of hospital stay.

## Data Availability

All data are available upon reasonable request to the corresponding author.
